# Application of MRI Image Based on Computer Semiautomatic Segmentation Algorithm in the Classification Prediction of Breast Cancer Histology

This article has been retracted.

**DOI:** 10.1155/2021/6088322

**Published:** 2021-11-24

**Authors:** Aizhu Sheng, Aijing Li, Jianbi Xia, Yizhai Ye

**Affiliations:** ^1^Hwa Mei Hospital, University of Chinese Academy of Sciences, Ningbo Institute of Life and Health Industry University of Chinese Academy of Sciences, Ningbo, Zhejiang 315010, China; ^2^Ninghai First Hospital, Ningbo, Zhejiang 315600, China

## Abstract

**Objective:**

The study aimed to investigate the predictive classification accuracy of computer semiautomatic segmentation algorithm for the histological grade of breast tumors through the magnetic resonance imaging (MRI) examination.

**Methods:**

Five dynamic contrast-enhanced (DCE) MRI regions of interest (ROIs) were captured using computer semiautomatic segmentation method, referring to the entire tumor area, tumor border area, proximal gland area, middle gland area, and distal gland area. According to the mutual information maximum protocol, the corresponding five ROIs were extracted from diffusion weighted imaging (DWI) combined with DCE-MRI images. To use the features in the nonoverlapping area of DWI image and DCE-MRI image as elements, a single-variable logistic regression model was established corresponding to element characteristics. After multiple training, the model was evaluated using the receiver operating characteristic (ROC) curve and area under curve (AUC).

**Results:**

This DCE-MRI combined with DWI was superior to DCE-MRI and DW in the prediction of tumor area features. To use DCE-MRI or DWI alone was less effective than DCE-MRI combined with DWI. The DWI combined DCE-MRI demonstrated good regional segmentation effects in the tumour area, with luminal A value being 0.767 and the area under curve (AUC) value being 0.758. After optimization, the AUC value of the tumor area was 0.929, indicating that classification effects can be enhanced by combining the two imaging methods, which complemented each other.

**Conclusions:**

The DWI combined DCE-MRI imaging has improved the early diagnosis effects of breast cancer by predicting the occurrence of breast cancer through the labeling of biomarkers.

## 1. Introduction

Under tremendous pressure for breast cancer treatment [1], it is desperately needed to prevent breast cancer through deep learning of a large amount of clinical individual data, together with the optimization of tumor detection methods according to tumour molecular characteristics [2]. MRI can detect concealed lesions, and drug treatment in the early stage can exempt the patient from the resection surgery in the advanced stage [3]. For patients who are diagnosed with breast cancer for the first time, the disease condition is classified through image detection. Based on different imaging parameters, there are DCE-MRI imaging and DWI imaging [4–6], displaying distinct tumour histological characteristics. DCE-MRI mainly presents the morphological characteristics of the lesion. DWI is able to perform detection in vivo using microscopic motion imaging of water molecules. They are usually used in combination to diagnose breast cancer [7].

To segment the boundaries of breast cancer tissue based on the personal experience of the radiographer and computer analysis technology, the image segmentation is greatly sped up [8, 9]. The histopathological classification of breast cancer is closely associated with breast cancer treatment and postoperative recovery. A higher histopathological grade of breast cancer indicates a higher failure rate of early clinical treatment, which can be attributed to that the tumor is more prone to spread. To identify the histological grade in time and determine a more suitable treatment method is beneficial to the diagnosis and treatment of breast cancer [10, 11].

Based on this, this paper proposed a computer semiautomatic segmentation method to collect five dynamic enhanced MRI areas of interest (ROIs), including the whole tumor area, the marginal tumor area, the proximal glandular area, the middle glandular area, and the distal glandular area. According to the maximum mutual information protocol and combined with DCE-MRI images, the corresponding five ROIs were extracted from DWI. The features of nonoverlapping regions of DWI images and DCE-MRI images were used as elements to establish a univariate logistic regression model corresponding to element features.

## 2. Materials and Methods

### 2.1. Clinical Data

A total of 116 female breast cancer patients hospitalized from May 2018 to May 2020 were selected as the research subjects. Inclusion criteria: (i) patients diagnosed with invasive cancer by pathological examination through hollow needle aspiration; (ii) patients who had the MRI examination for the breast; (iii) the treatment time in the hospital was more than 4 weeks. Exclusion criteria: (i) patients with incomplete clinical data; (ii) patients with clinical treatment less than 4 weeks due to personal reasons; (iii) patients who did not receive MRI examination; (iv) patients with other system diseases; (v) patients who transferred from other hospitals. After screening by the above criteria, 68 people were finally identified. They were 28–69 years old, with an average age of 47.11 ± 9.59 years and a median age of 47.

### 2.2. MRI Examination

The SIEMENS Verio 3.0 T magnetic resonance was applied, and a 4-channel breast phased array coil was used for image acquisition. During the examination, the patient remained prone, so that the breasts on both sides hang naturally in the center of the coil. The axial, sagittal, and coronal images were obtained. The short-time inversion recovery (STIR) sequence (TR 4300 ms, TE 61.0 ms, layer thickness 4 mm, FOV 340 mm × 340 mm) scanning axial 3D FLASH T1 sequence scanning (TR 6.05 ms, TE 2.46 ms, layer thickness 1.3 mm, FOV 340 mm × 340 mm) was performed sequentially. Once the DCE-MRI scan was finished, T1 sequence delayed scan (TR 8.75 ms, TE 4.33 ms, slice thickness 0.9 mm, FOV 340 mm × 340 mm), conventional T2 axial scan (TR 4500 ms, TE 79 ms, slice thickness 4.0 mm, FOV 340 mm × 340 mm), and DWI scanning (*b* = 800 s/mm^2^, TR 7200 ms, TE 74 ms, layer thickness 4.0 mm, FOV 380 mm × 380 mm) were performed immediately.

### 2.3. Clinical Data Statistics

The clinical information was sorted out, including age, tumor histological grade, estrogen receptor (ER) content, progesterone receptor (PR) content, and changes in the expression levels of HER-2 and Ki-67. The subtypes of tumor cells were identified according to the results of H&E staining.

The identification protocol was as follows. (i) Luminal A : ER/PR (+) and high expression of PR, HER-2 (−), Ki 67 < 14%. (ii) Luminal B : ER/PR (+), HER-2 (−), Ki67 ≥ 14%; or ER/PR (+), HER-2 (+). (iii) Triple-negative breast cancer (TNBC) : ER/PR (−), HER-2 (−). (iv) HER-2 type: ER/PR (−), HER-2 (+).

### 2.4. Multiparameter MRI Analysis

The ITK snap (version: 3.8.0-beta; https://www.itksnap.org) software was used to preprocess MRI images. The T1 image was taken 90 s after the injection of the contrast agent, and the identification of ROI and the volume of interest (VOI) were determined. The cancer tissue can be distinguished from normal tissue by comparing the background enhancement degree. Because that of the lesion reached its peak, while in normal tissue, the background enhancement was weaker. The steps for processing the ROI were as follows. An imaging doctor manually outlined the ROI layer by layer, and then another doctor revised the outlined area. If there was a controversial area, a final assessment was made under discretion of a third doctor with more clinical experience. A 3D VOI was finally identified following unanimous results from the three doctors (Figure 1). The outlined VOI should include all cystic necrosis areas, derived peripheral burrs, and surrounding blood vessels and fibrous tissues. The operation process is shown in Figure 2.

Artificial intelligence medical big data image cloud platform (Huiyi Huiying) was used to capture 1029 image features from the acquired VOI (Table 1), which were divided into 4 categories of shape- and size-based features, texture features, first-order statistics, and higher order statistics features.

The least absolute shrinkage selection operator (LASSO) was used to reduce the feature dimension to gradually select the most effective optimization features. The 10-fold cross-validation method was used to find the best alpha value in the sequence, and the coefficients of different properties corresponding to the alpha value were then selected, followed by the identification of the function if the coefficient was not 0. The most relevant features obtained are shown in Figure 3.

The data were divided into two categories at a ratio of 8 : 2, which were the training set containing 57 samples and the test set containing 16 samples. The input eigenvalues were then standardized to improve prediction ability. The logistic regression (LR) was applied to classify features, and the ROC curve was used to evaluate the prediction effect of the model. The optimal cutoff value was obtained based on maximum Yoden index (sensitivity + specificity − 1). Subsequently, it was verified whether the two cutoff values were consistent. The AUC value, sensitivity, specificity, accuracy, and F1 score were calculated according to the ROC of the training set and the test set, followed by evaluation of the prediction effect of the model.

## 3. Results

### 3.1. Feature Analysis of the DCE-MRI Image of the Tumor Area

There were a total of 87 features extracted from DCE-MRI images, including 19 texture features, 10 statistical features, and 58 dynamic enhancement features. The single-variable regression was performed with 87 features as independent variables and breast cancer grade and molecular typing labels as dependent variables. At the same time, two classification models were trained using Luminal A and non-Luminal A; Luminal B and non-Luminal B; HER-2 and non-HER-2; and basal-like and non-basal-like for the prediction molecular typing labels. The leave-one-out cross-validation method was used to evaluate the prediction effect based on the AUC value. The optimal features were recorded, as shown in Table 1.

It was evident from the table that, after sorting each tag, the first three AUC functions listed in the table are used as tags for checking. Except for the maximum value, the degree of deviation (two choices) and the range belonging to statistical features, the other attributes were generated by the mask sequence to include all the texture attributes of the two gray-scale difference sequences S3–S0 and S5–S0. The above information illustrated that the texture feature of the above labels exhibited higher resolution versus the statistical feature. In the classification of Luminal A and non-Luminal A, the highest AUC value reached 0.642 from S5–S0. In the classification of Luminal A and non-Luminal, the AUC value of the single feature was higher than that of other label classification methods. The features in Table 2 were all the texture features of dynamic enhancement, which indicated that the DCE- MRI played an important role in tumor label prediction of breast cancer.

### 3.2. The DWI Image Feature Analysis in the Tumour Area

The same method was used to evaluate the prediction effects of a single feature on the label in the tumour area using DWI, and the results are shown in Table 2.

It was evident that the texture features demonstrated relatively good prediction effects for historical grade and Luminal A, and there was only one statistical feature. There were few differences in prediction effects of selected labels between DCE-MRI features and DWI features. As with DCE-MRI, after the binary classification of Luminal A, the AUC values of the top three single features were relatively overall higher. With features obtained by classifying Luminal A under DCE combined with MRI as reference, the features of DWI showed better prediction effects, indicating that DWI had better performance in predicting breast cancer biomarkers at an early stage.

### 3.3. Univariate Prediction Effect of Histological Grade

As shown in Table 3, the DCE-MRI and DWI showed no notable difference in the prediction of histological grade. The features with better prediction effects came from the tumor area or S-B and S-T areas. Taken together, these results indicated that taking tumor boundaries and tissue around the glands as biomarkers had important functions in predicting the occurrence of breast cancer.

### 3.4. Analysis of Multivariate Prediction Results

The classification results are shown in Figure 4 after feature fusing and selection of AUC as the reference index.

For DCE-MRI, histological grade, Luminal A, and HER-2 basal-like were 0.7, 0.82, 0.39, and 0.58, respectively. Histological grade, Luminal A, and HER-2 basal-like were 0.64, 0.8, 0.68, and 0.65, respectively. Histological grade, Luminal A, and HER-2 basal-like were 0.78, 0.92, 0.74, and 0.75 for DCE-MRI combined with DWI. It was found that DCE-MRI combined with DWI was superior to DCE-MRI and DW in the prediction of tumor area features. Using DCE-MRI or DWI alone was less effective than DCE-MRI combined with DWI. Also, it suggested that imaging parameters of different attributes can be fused.

This paper introduces the application of a knowledge-based segmentation method in automatic detection of follicular outer wall boundary in an ovarian ultrasound image. Combining computer detection and interactive adjustment, the approximate inner wall boundary of follicle was defined, and then the outer wall boundary of the follicle was automatically searched by computer algorithm as a prior knowledge [12].

## 4. Conclusion

According to the tumor area in DCE-MRI and DWI images, the biomarker of breast tumor was predicted. DWI images and breast fibrous tissue with different information were used as the follow-up test subjects of DCE-MRI to explore the prediction effects of biomarkers on the breast cancer grade. Patients who met the requirements were selected after screening, followed by the analysis of their DCE-MRI and DWI images. Many subregions of interest were then obtained using computer segmentation algorithms, from which a series of statistical features, texture features, and dynamic enhancement features were extracted, followed by the construction of the classifier model based on different feature selection methods. Subregion images with different display parameters were analyzed to compare the prediction effects. The results showed that there was no notable difference in the prediction effects of DWI and DCE-MRI for tumor biomarkers. At the same time, they complemented each other in terms of features contained in different imaging parameters.

The existing experimental results revealed that the classification effects of the constructed model on Luminal B features were not as good as expected. The reason for this may be that the features extracted were not enough [13–15]. In the follow-up experiments, based on the biological features of Luminal B tumors, it is needed to obtain other new features from the images and incorporate new features into the artificial intelligence big data to improve prediction accuracy, so as to provide a theoretical basis for breast cancer diagnosis.

## Figures and Tables

**Figure 1:** The segmentation of 3D VOI.

**Figure 2:** Breast tumor segmentation flowchart.

**Figure 3:** Model construction flowchart.

**Figure 4:** Multivariate prediction results of tumor.

**Table 1:** The optimal single feature in DCE-MRI image of the tumor area.

Label	Feature name	AUC				
Histological grade	Deficit	Square gap	Contrast	0.623	0.629	0.631
Luminal A	Difference entropy	Not similar	Contrast	0.639	0.642	0.622
Luminal B	Autocorrelation	Cluster shadow	Skewness	0.607	0.614	0.616
HER-2	Related information test	Max	Very bad	0.589	0.604	0.613
Basal-like	Skewness	Squared variance	Autocorrelation	0.627	0.592	0.606

**Table 2:** The optimal single feature of DWI image in the tumour area.

Label	Feature name	AUC
Histological grade	And average	0.628
	Sum of squares of variance	0.637
	Cluster shadow	0.641
Luminal A	Related information measures	0.767
	Related information measures	0.731
	Max	0.758

**Table 3:** High AUC value areas and the top three features in the prediction of histological grade.

DCE-MRI	Feature name	AUC	DWI	Feature name	AUC
S-T	Deficit^1^	0.623	S-T	Sum of squares of variance	0.637
	Square gap^2^	0.629		And average	0.628
	Contrast^2^	0.631		Cluster shadow	0.641
S-B	Correlation^3^	0.613	S-B	Correlation	0.635
	Cluster shadow^2^	0.628		Entropy	0.627
	Difference entropy^3^	0.630		And entropy	0.642

## Data Availability

The data used to support the findings of this study are available from the corresponding author upon request.
